# A Nanoparticle-Conjugated Anti-TBK1 siRNA Induces Autophagy-Related Apoptosis and Enhances cGAS-STING Pathway in GBM Cells

**DOI:** 10.1155/2021/6521953

**Published:** 2021-12-11

**Authors:** Shengchao Xu, Xi Yan, Lu Tang, Gan Dai, Chengke Luo

**Affiliations:** ^1^Department of Neurosurgery, Xiangya Hospital of Central South University, Changsha 410008, Hunan, China; ^2^National Clinical Research Center for Geriatric Disorders, Xiangya Hospital, Central South University, Changsha, China; ^3^Health Management Center, Xiangya Hospital of Central South University, Changsha 410008, Hunan, China; ^4^Department of Thoracic Surgery, Xiangya Hospital of Central South University, Changsha 410008, Hunan, China; ^5^Department of Microbiology, School of Basic Medical Science, Central South University, Changsha 410008, China

## Abstract

**Background:**

Gene therapy shows considerable clinical benefit in cancer therapy, in which single-stranded ribonucleic acid (siRNA) is a promising strategy in the treatment of glioblastoma (GBM). TANK-binding kinase 1 (TBK1) is critical in tumorigenesis and development, which lays a foundation for an ideal target for tumor therapy. However, the practical application of free siRNA is limited. It is urgent to develop novel strategies to deliver TBK1 siRNA to activate apoptosis and cGAS-STING pathway as a therapeutic strategy for GBM.

**Methods:**

The expression and prognostic value of TBK1 were evaluated in the TCGA, CGGA, and GTEx databases. A novel gene delivery system was designed here via PEGylated reduced graphene oxide (rGO-PEG) to targeted delivery of anti-TBK1 siRNA efficiently. The efficacy of TBK1si/rGO-PEG was evaluated in GBM cells. The underlying pathways were explored by Western blot.

**Results:**

TBK1 was highly expressed in glioma samples, and its high expression indicated poor prognoses in glioma patients. The rGO-PEG presented great efficiency in targeted delivery of TBK1si RNA into GBM cells with up to 97.1% transfection efficiency. TBK1si/rGO-PEG exhibited anti-GBM activities by inhibiting TBK1 and autophagy, as well as activating apoptosis and cGAS-STING pathway.

**Conclusion:**

The rGO-PEG could be an efficient system facilitating the delivery of specific siRNA. TBK1si/rGO-PEG could be a novel strategy for the treatment of GBM.

## 1. Introduction

The incidence of glioblastoma (GBM, grade IV) in Western countries and China is increasing year by year, which owned the highest mortality rate [1, 2]. Some biomarkers such as isocitrate dehydrogenase (IDH) mutation and 1p19q codeletion have been proposed to indicate favorable prognosis of glioma patients [3, 4]. Besides, age is considered as a prognostic factor for glioma patients, and the younger age indicates a favorable prognosis [5, 6]. The conventional therapies include surgery, chemotherapy, and radiotherapy; however, the average survival time of GBM patients ranges from 12 to 15 months [7, 8]. Although gene regulation is regarded as a key factor for tumorigenesis, the application of gene therapy remains controversial. Hence, the treatment for GBM is challenging.

TANK-binding kinase 1 (TBK1) is a noncanonical member of the inhibitor of nuclear factor *κ*B (IKK) family, which is involved in cell survival, autophagy, mTOR/AKT signaling, and KRAS-driven tumorigenesis [9, 10]. Moreover, EGFR constitutively complexes with TBK1 and leads to TBK1 phosphorylation in glioblastoma [11]. The loss of TBK1 inhibits kidney cancer cell growth [12]. Therefore, downregulation of TBK1 may be a promising approach to suppress the progression of GBM, which has not been reported yet.

As an emerging and promising tool, gene therapy has attracted increasing attention in the treatment of cancers or autoimmune diseases [13]. RNA interference (RNAi), a conserved biological response to double-stranded RNA, is about 20–25 nucleotides, which binds to the specific target gene to manipulate gene expression by inhibiting mRNA and protein. As variously known, siRNA can regulate gene expression specifically, which is essential in RNAi phenotype. SiRNA may be a promising strategy in the treatment of cancers including GBM. However, the practical application of free siRNA is limited, owing to the inefficient cellular uptake and nuclease degradation because of its enzyme vulnerability and negative charges. Consequently, it is urgent to modify siRNA and make it used more widely, especially in GBM.

Based on our previous work [14], graphene oxide (GO) can stabilize proteins. From this, we further designed TBK1si/rGO-PEG to targeted delivery of TBK1si RNA into GBM cells. This work may facilitate and expand the experimental, even clinical applications of siRNA in targeted therapy.

## 2. Materials and Methods

### 2.1. Data Extraction

The expression of TBK1 in gliomas and normal brain tissues was extracted from The Cancer Genome Atlas (TCGA), Chinese Glioma Genome Atlas (CGGA), and Genotype-Tissue Expression (GTEx) databases. A total of 672 and 1013 glioma patients were included in the TCGA and CGGA datasets, respectively. GEPIA website was used to detect the expression of TBK1 in gliomas and normal brain tissues [15].

### 2.2. Subgroup Analysis

For subgroup analysis, patients were divided into two groups based on the following variables: grade (III or IV), IDH status (wildtype or mutant), and age (≤41 years old or >41 years old).

### 2.3. Characterization of rGO-PEG Nanoparticles

For GO functionalization, 2 mg of GO was diluted in 2 ml ultrapure DI (Deionized) water and then added 20 mg PEG-NH2. Put those mixtures under sonication for 90 min. Then, the mixture was mixed with 20 mg EDC and stirred for 12 h. Afterward, centrifuged at 20000 rpm for 30 min to remove excess free PEG-NH2. At last, resuspended the precipitate into 2 mL ultrapure DI water. The rGO-PEG was synthesized in the presence of GO-PEG and NaBH4. Last, rGO-PEG with the final concentration of 2 mg/mL was achieved after centrifugation to remove excess free reagents.

The TBK1si/rGO-PEG was diluted with distilled water, put on a copper grid with nitrocellulose, and then stained with phosphotungstic acid. Afterward, it was measured by Nano ZS-90 (Malvern Instruments, Malvern, UK) under room temperature. AFM (atomic force microscopy) images were taken by a Nanoscope V multimode atomic force microscope (Veeco Instruments, USA). TBK1si/rGO-PEG was diluted with ultrapure DI water with a final concentration of 1 × 10^−6^ M for AFM. Twenty *μ*L TBK1si/rGO-PEG sample was placed on the brand new muscovite mica and dried the samples under critical point dryer. Photos were taken in the tapping mode under room temperature.

### 2.4. Preparation of TBK1si/rGO-PEG Complexes

For siRNA loading, single-chain anti-TBK1 siRNA (TBK1si) was dispersed in ultrapure DI water. TBK1 siRNA (20 nM) in 1 mL ultrapure DI water was added into rGO-PEG (2 mg/mL). Those samples were mixed and stirred for half a day at 37°C. Then, samples were centrifugated to remove free TBK1si. The TBK1si/rGO-PEG nanoparticles ranging 5 : 1, 50 : 1, and 500 : 1 (weight ratios, siRNA: rGO-PEG) were electrophoresed under 150 V for half an hour. Then, the agarose gel was stained and illuminated to show the blot of RNA.

### 2.5. Cell Transfection

The U251 cells, purchased from American Type Culture Collection (Manassas, VA, USA), were cultured in six-well plates at the density of 2 × 10^5^/well with 4 mL complete DMEM for a day. Then, the medium was changed to fresh serum-free DMEM while transfection. Fluorescein isothiocyanate (FITC)-labeled TBK1si (TBK1si-FITC) was designed and the quantity of which was about at 0.1 nm/well. The weight ratios of TBK1si-FITC/rGO-PEG range 5 : 1, 50 : 1, and 500 : 1. To detect the transfected cells and evaluate the transfection efficiency, the fluorescence signal was measured by the LSR Fortessa device (BD Biosciences, San Jose, CA, USA) and the fluorescence microscope (Carl Zeiss Meditec AG, Jena, Germany). The Consi sequence was 5′-UUCUCCGAACGUGUCACTUTT-3′.

### 2.6. CCK8 Assay

A total of 1 × 10^4^ of U251 cells were seeded in 96-well plates. TBK1si/rGO-PEG were synthesized by TBK1 siRNA (TBK1si1: UAAACUUCUAUUAGAAAGCUA; TBK1si2: UGAACUGAUAGUAAAUCUCUG; TBK1si3: UAAUCUGCUGUCGAUAUCCUG), respectively. After incubation with NS (normal saline), rGO-PEG, Consi/rGO-PEG, or TBK1si/rGO-PEG for 3, 24, 48, and 72 h, 10 *µ*L CCK8 reagent was added into wells and cultured for 2 h. The absorbance at 450 nm was evaluated by the Bio-Rad reader to assess GBM cell viability.

### 2.7. Cell Cycle Analysis

GBM cells were cultured in 12-well plates at the density of 1 × 10^5^/well with 2 ml complete DMEM with 10% FBS. After 12 h, GBM cells were treated with NS, rGO-PEG, Consi/rGO-PEG, or TBK1si/rGO-PEG for 48 h. Then, all GBM cells were harvested and fixed in 70% ethanol for 12 h at 4°C. After washed twice by PBS, GBM cells were incubated RNase A for 1.5 h at room temperature. Afterward, propidium iodide (PI) (Becton–Dickinson, San Jose, CA) and Triton X-100 were used to stain GBM cells. At last, the LSR Fortessa device (BD Biosciences, San Jose, CA, USA) was used to acquire the data, which were analyzed with FlowJo V10.

### 2.8. Cell Apoptosis Analysis

GBM cells were cultured in six-well plates at a density of 1 × 10^5^ cells/well with 4 ml complete DMEM for 12 h. Then, GBM cells were treated with NS, rGO-PEG, Consi/rGO-PEG, or TBK1si1/rGO-PEG for 12 h. Afterward, the cells were collected and stained by the Annexin V-CF Blue/PI apoptosis detection kit (Abcam) as protocol for 20 min at 25°C in the darkness. The LSR Fortessa device (BD Biosciences, San Jose, CA, USA) was used to evaluate the apoptotic cells including the early and late ones in GBM cells.

### 2.9. Western Blotting

The GBM cells washed with cold PBS were lysed with radioimmunoprecipitation assay buffer (ThermoFisher) containing phenylmethyl sulfonylfluoride (Sigma-Aldrich) and protease inhibitor cocktail (Cell Signaling). Then, the supernatant was collected, and the protein could be measured roughly after the lysate was centrifuged. After electrophoresed on a 10% SDS-PAGE gel at 120 V for 60 min, proteins were transferred onto Immobilon PSQ PVDF membranes (ThermoFisher) at 100 V for another 60 min. After blocked in membrane blocking solution (Invitrogen) for 1 h at 25°C, blot was mixed with primary antibodies for 12 h at 4°C, which was tested by the corresponding horseradish peroxidase-conjugated secondary antibody. It was incubated with the Pierce ECL kit (SignaGen, Jinan, China). Antibodies include rabbit anti-TBK1 (1 : 1,000 dilution; CST, Boston, MA, USA), *β*-actin (Clone 13E5; Cell Signaling, #4970, 1 : 2000), STING (Clone D2P2F; Cell Signaling, #13647, 1 : 500), and cGAS (Clone D3O8O; Cell Signaling, #31659, 1 : 500) goat anti-rabbit IgG antibody (1 : 5,000 dilution). The critical molecules in partway were probed with primary antibodies against caspase-3, Bcl-2, P53, P62, p-P62, p-TBK1, cGAS, STING, and LC3.

### 2.10. Statistical Analyses

The data were analyzed and visualized by R version 3.6.0 and GraphPad Prism version 8.0.2. Kaplan–Meier analysis was used to estimate the survival difference between TBK1-high and TBK1-low groups. The optimal cutoff point of TBK1 expression in survival analysis was determined using “survminer” R package. Statistical analysis was accessed by the unpaired two-tailed Student's *t*-test or one/two-way ANOVA variance. All data were shown as mean ± standard deviation. Asterisks indicated the various statistical significance (^*∗*^*p* < 0.05, ^*∗∗*^*p* < 0.01, ^*∗∗∗*^*p* < 0.001). n.s. means nonsignificant, indicating *p* > 0.05. Error bar = mean ± standard deviation presented in all necessary graphs.

## 3. Results

### 3.1. TBK1 Was Highly Expressed in Gliomas and Correlated with the Prognosis of Glioma Patients

To preliminarily explore the potential role of TBK1 in gliomas, we extracted data from online databases including TCGA, CGGA, and GTEx. The expression of TBK1 was significantly elevated in lower-grade glioma (LGG, grade II and III gliomas) and GBM compared with normal brain tissues (*p* < 0.05) (Figure 1(a)). Glioma patients with low expression of TBK1 had relatively better survival time compared with those with high TBK1 expression (*p* < 0.05) (Figure 1(b)). In subgroup analysis, the low expression of TBK1 indicated better prognoses for patients with grade III or IV glioma (*p* < 0.05) (Figures 1(c) and 1(d)). Moreover, in IDH wildtype or mutant glioma patients, those with low expression of TBK1 had a relatively long overall survival time (*p* < 0.05) (Figures 1(e) and 1(f)). These findings were consistent in glioma patients who were younger than 41 years old or not (*p* < 0.05) (Figures 1(g) and 1(h)). These results indicated that TBK1 played a potential carcinogenic role in glioma and correlated with the prognosis of glioma patients.

### 3.2. Preparation and Characteristics of TBK1si/rGO-PEG

GO was obtained according to our previous work [14, 16] in the presence of EDC and conjugated with six-arm PEG into GO-PEG [17]. Then, GO-PEG was reduced by NaBH4 with rGO-PEG yielded. It is critical to raise the chemistry and physiological stability of rGO or GO via PEG functional modification. rGO-PEG absorbed siRNA and consisted of TBK1si/rGO-PEG, with a sheet shape (Figure 2(a)). rGO-PEG significantly improved the stability with the culture medium, which was similar to physiological conditions (Figure 2(b)). The average diameter of the miRNA-loaded nanoparticles was 102.00 ± 20.53 nm, and the height of TBK1si/rGO-PEG is 18.00 ± 3.18 nm in AFM image (Figures 2(c) and 2(d)). The UV–vis absorption spectrum revealed that after the alternation from GO-PEG into rGO-PEG, the absorption maximum presented a significant redshift from 230 nm to 265 nm, but there was no 265 nm nearby peak for PEG (Figure 2(e)). Those results indicated that the redshift of the UV spectrum was on the basis of the restoration of electronic conjugation in the rGO, instead of the existence of PEG [17].

### 3.3. Stability and Release Rate of TBK1si/rGO-PEG

The fluorescence emission spectrum was measured after the TBK1si/rGO-PEG nanoparticles were mixed with a certain concentration (1 *μ*M) of complementary DNA. Only 20% of the labeled TBK1si released from rGO-PEG to complete DMEM after 3 d (Figure 3). However, over 70% of the TBK1si is released in the presence of corresponding complementary dye-labeled siRNA within 10 h (*p* < 0.05). This result could lay a solid foundation of a brand new and efficient platform based on siRNA/rGO-PEG nanoparticles for targeting the gene in vitro and even in vivo.

### 3.4. Transfection Efficiency and Its Effects of TBK1si/rGO-PEG In Vitro

The TBK1si-FITC/rGO-PEG was prepared in various weight ratios ranging 5 : 1, 50 : 1, and 500 : 1. After incubation with TBK1si-FITC/rGO-PEG in three different ratios for 3 h, the GBM cells transfected by the ratio of 500 : 1 exhibited the brightest fluorescence under fluorescence microscopy (Figure 4(a)), indicating the highest transfection efficiency. After evaluated by flow cytometry, the transfection efficiency of three different ratios ranging 5 : 1, 50 : 1, and 500 : 1 was 72.2%, 90.8%, and 97.1%, respectively (Figure 4(b)). In order to suppress the expression of TBK1, GBM cells were transfected with NS, rGO-PEG, Consi/rGO-PEG, TBK1si1/rGO-PEG, TBK1si2/rGO-PEG, and TBK1si3/rGO-PEG. After 48 h of transfection, the expression of TBK1 was decreased the most in the TBK1si1/rGO-PEG treatment group than other groups (*p* < 0.001) (Figures 4(c) and 4(d)).

### 3.5. TBK1si/rGO-PEG Inhibited Proliferation and Induced Apoptosis of GBM Cells

GBM cell viability was investigated by CCK8, which presented that the viability in the TBK1si1/rGO-PEG group was significantly lower than other control groups (*p* < 0.05) (Figure 5(a)). Moreover, representative images reflected the effect of NS, rGO-PEG, Consi/rGO-PEG, and TBK1si/rGO-PEG (Figure 5(b)). TBK1si1/rGO-PEG nanoparticles induced cell cycle arrest in the G1/S phase more significantly than any other interventions (Figure 5(c)). At last, the apoptosis rate was evaluated with Annexin V/PI kit by flow cytometry. The apoptosis rates of NS, rGO-PEG, Consi/rGO-PEG, or TBK1si/rGO-PEG groups were 0.85%, 0.33%, 1.40%, and 47.50%, respectively (Figure 5(d)). TBK1si/rGO-PEG significantly induced cell apoptosis compared with other interventions (*p* < 0.05) (Figure 5(e)).

### 3.6. TBK1si/rGO-PEG Inhibited Autophagy but Activated cGAS-STING Pathway

To reveal the mechanism of the anti-GBM effect of TBK1si/rGO-PEG, the critical protein expression level of apoptosis and autophagy after the interventions of NS, rGO-PEG, Consi/rGO-PEG, or TBK1si/rGO-PEG were measured. In Figure 6(a), Bcl-2 and caspase-3 expressions were dropped, and P53 enhanced after the treatment of TBK1si/rGO-PEG, pointing that this nanoparticle may be induced by apoptosis via the P53 pathway. Afterward, the expression of cGAS, STING, LC3, p-TBK1, and p-P62 after TBK1si/rGO-PEG treatment was also tested (Figure 6(b)). The result presented that p-TBK1, LC3-II, and p-P62 significantly decreased and cGAS, STING, P62, and LC3-I increased after 3 days of treatment with TBK1si/rGO-PEG, whereas TBK1 and *β*-actin were not affected.

## 4. Discussion

Gene regulation plays a critical role in the development of cancer including cell proliferation, angiogenesis, immunology, and metastasis. The gene mutations can lead to tumorigenesis [18–21]. However, the treatment of malignant tumors including GBM remains a challenge. Gene therapy is promising for the treatment of cancer and certain autoimmune diseases [22–25]. Particularly, gene was transferred into the abnormal cell to produce a functional molecular, such as protein, which can correct a genetic disorder [26–29].

TBK1 and its I*κ*B kinase epsilon (IKK*ε*) are noncanonical members of the IKK family. Their roles in innate immune signaling and cancer have been well characterized, including promotion of cell survival, autophagy, and AKT–mTOR signaling, and TBK1 activation promotes KRAS-driven tumorigenesis and development [9, 10]. Furthermore, TBK1 signaling in both cancer and immune cells can promote immunosuppression, and potent/specific TBK1 inhibitors have been shown to potentiate ICI responsiveness in preclinical models [10, 30]. TBK1 also activates type-1 IFN signaling downstream of the cGAS-STING pathway and other viral and pathogen sensors and thus can regulate both pro and antitumorigenic innate immune pathways [31]. Moreover, EGFR constitutively complexes with TBK1 leading to TBK1 phosphorylation in glioblastoma [11]. Based on those points, inhibition of TBK1 could obviously prevent GBM from proliferation. TBK1 could be inhibited by various methods such as siRNA, shRNA, or inhibitors. The transfection efficiency of shRNA is low since it is a plasmid system, which is hard to deliver via a nonviral vector. Although the transfection efficiency could be enhanced by a viral vector system, the safety issue should be addressed. In addition, small-molecule inhibitors are limited for its specificity, in spite of being focused recently. As a result, the siRNA is more promising for its safety and reliability in nonviral vector transfection. Due to the specific properties such as enzyme vulnerability and negative charges, siRNA is limited in application for inefficient cellular uptake and nuclease degradation. Thus, it is urgent to develop novel strategies for transporting siRNA. The virus system and physical methods are popular, but the delivery and security issues should be addressed [32, 33]. Since the 1960s, many chemical transfection systems including calcium phosphate, lipid, and cationic polymers have been designed as an alternative to viral vectors to overcome the previous shortcomes [24, 34]. Afterward, many efforts have been devoted to modify chemical molecular features such as structure, size, and surface potential to enhance the transfection efficiency [35, 36]. However, the ideal siRNA delivery system should possess not only high transfection efficiency but also low toxicity. Therefore, TBK1si/rGO-PEG was designed to inhibit TBK1 for GBM treatment. First, three different target RNA sequences were synthesized to inhibit the TBK1 protein expression, and results presented that TBK1si1 was the most efficient. Second, TBK1si1 was used to evaluate the anti-GBM effect. Those results presented that TBK1si1/rGO-PEG could significantly impede the proliferation of GBM than other groups including NS, rGO-PEG, Consi/rGO-PEG, and TBK1si/rGO-PEG. As a result, the TBK1si1/rGO-PEG nanoparticle was used as the target delivery system for TBK1 siRNA.

In this study, autophagy-related molecular expression was investigated, and the result presented that inhibition of TBK1 can upregulate the expression of caspase-3, P53, P62, LC3-I, cGAS, and STING, while downregulating the Bcl-2, p-TBK1, p-P62, and LC3-II. Therefore, we found that TBK1siRNA promotes apoptosis via inhibiting autophagy probably. Meanwhile, the damaged DNA activated P53, which results in cell cycle arrest and apoptosis. As is known, autophagy can be inhibited by the knockdown of TBK1, which lays a foundation of accumulation of P62. Interestingly, the cGAS-STING pathway was enhanced probably by the accumulation of P62 [37], which could promote the cell survival or initiate resistance in the presence of damage or medicine [31]. The cGAS-STING pathway is an evolutionary conserved defense mechanism against viral infections. It is reported that activation of TBK1 and cGAS-STING resulted in cancer progression and inflammation [38]. In cancers, it remains unclear how cGAS-STING axis suppresses type-1 IFN signaling and upregulate NF-*κ*B pathways to enhance metastatic behaviors. Maybe, the intensity of cGAS-STING activation determinates the switch between tumor suppression or promotion [39]. Yet, the underlying mechanisms remain poorly understood and require further research. The shortcomings in our work should be addressed, the possible mechanism of anti-GBM needs to be further studied, and TBK1si/rGO-PEG needs to be further studied whether it can effectively inhibit GBM growth in vivo.

## 5. Conclusions

The rGO-PEG could be an efficient system for the delivery of siRNA, and TBK1si/rGO-PEG could be a novel therapeutic approach for GBM treatment.

## Figures and Tables

**Figure 1:** TBK1 was highly expressed in gliomas and correlated with the prognosis of glioma patients. (a) The expression of TBK1 in lower-grade glioma (LGG) and glioblastoma (GBM) compared with normal brain tissues. (b) Kaplan–Meier analysis of TBK1 in glioma patients in the TCGA and CGGA datasets. (c)–(h) Kaplan–Meier analysis of TBK1 in grade III (c), grade IV (d), IDH wildtype (e), IDH mutant (f), ≤41 years old (g), or >41 years old (h) glioma patients in the TCGA and CGGA datasets. ^*∗*^*P* < 0.05.

**Figure 2:** The characteristics of TBK1si/rGO-PEG. (a) The rGO-PEG was prepared and (b) more stable than GO in RPMI1640 with 10% FBS. (c) Size distribution measured by Malvern Zetasizer Nano ZS-90 of TBK1si/rGO-PEG. (d) AFM image of TBK1si/rGO-PEG. (e) UV–vis absorption spectrum of rGO, PEG, and rGO-PEG. The result was a representative of three independent experiments.

**Figure 3:** Stability and release rate of TBK1si/rGO-PEG. Release behavior of TBK1si from rGO-PEG after addition into complete medium and complementary DNA, respectively. The result was a representative of three independent experiments. The *p* values were determined by the paired-samples *t*-test analysis. ^*∗∗∗*^*P* < 0.001.

**Figure 4:** Transfection efficiency of TBK1si/rGO-PEG and the expression of TBK1. TBK1si/rGO-PEG was used to transfect U251 cells for 3 hours. The transfection efficiencies at different weight ratios. (A) NS control and rGO-PEG vs. TBK1si as 1 : 5 (B), 1 : 50 (C), and 1 : 500 (D) accessed by the fluorescence microscope (a) and flow cytometry (b). When U251 cells were transfected with NS, rGO-PEG, Consi/rGO-PEG, or TBK1si/rGO-PEG for 3 days, TBK1 was investigated by RT-PCR (c) and Western blot (d). NS, normal saline. The result was a representative of three independent experiments. *P* values were determined by one-way analysis of variance (ANOVA) followed by Tukey post hoc test. ^*∗∗∗*^*P* < 0.001.

**Figure 5:** TBK1si/rGO-PEG exerted antitumor effects in vitro. (a) CCK8 analysis cell viability. When U251 cells were transfected with NS, rGO-PEG, Consi/rGO-PEG, or TBK1si/rGO-PEG for 3, 24, 48, and 72 hours, cell viability was tested by the CCK8 test. (b) Cell cycle analysis of U251 cells after 48-hour intervention with TBK1si/rGO-PEG. (c) Percentage of U251 cells in each mitotic phase after treatment with NS, rGO-PEG, Consi/rGO-PEG, or TBK1si/rGO-PEG. (d)-(e) When U251 cells were transfected with NS, rGO-PEG, Consi/rGO-PEG, or TBK1si/rGO-PEG for 72 hours, U251 cells were collected and stained with Annexin V-CF Blue/PI and then analyzed by flow cytometry. Statistics of GBM cell apoptosis. PI, propidium iodide. The result was a representative of three independent experiments. Error bars represent mean ± SD. *P* values were determined by one-way analysis of variance (ANOVA) followed by Tukey post hoc test. ^*∗*^*P* < 0.05. ^*∗∗*^*P* < 0.01. ^*∗∗∗*^*P* < 0.001.

**Figure 6:** TBK1si/rGO-PEG exhibited the anticancer effect via activating the cGAS-STING pathway. (a) The effect of TBK1si/rGO-PEG on apoptosis-related proteins. (b) The autophagy was inhibited, and cGAS-STING was enhanced by TBK1si/rGO-PEG.

## Data Availability

The data used to support the findings of this study are available from the corresponding author upon request.
